The article "Intelligent Wearable Devices Enabled Automatic Vehicle Detection and Tracking System with Video-Enabled UAV Networks Using Deep Convolutional Neural Network and IoT Surveillance" was published in 2022. Journal: J Healthc Eng.

# Intelligent Wearable Devices Enabled Automatic Vehicle Detection and Tracking System with Video-Enabled UAV Networks Using Deep Convolutional Neural Network and IoT Surveillance

**DOI:** 10.1155/2022/2592365

**Published:** 2022-03-28

**Authors:** A. R JayaSudha, Pankaj Dadheech, K. Ramalingeswara Prasad, S. Hemalatha, Meghna Sharma, Sajjad Shaukat Jamal, Daniel Krah

**Affiliations:** ^1^Department of Computer Applications, Hindusthan College of Engineering & Technology, Coimbatore, India; ^2^Department of Computer Science & Engineering, Swami Keshvanand Institute of Technology, Management & Gramothan (SKIT), Jagatpura, Jaipur, Rajasthan, India; ^3^Department of EEE, Lakireddy Bali Reddy College of Engineering (A), Mylavaram, Andhra Pradesh, India; ^4^Department of Computer Science and Engineering, Panimalar Institute of Technology, Chennai, Tamil Nadu, India; ^5^Department of Computer Science and Engineering, The NorthCap University, Gurugram, India; ^6^Department of Mathematics, College of Science, King Khalid University, Abha, Saudi Arabia; ^7^Tamale Technical University, Tamale, Ghana

## Abstract

The discipline of computer vision is becoming more popular as a research subject. In a surveillance-based computer vision application, item identification and tracking are the core procedures. They consist of segmenting and tracking an object of interest from a sequence of video frames, and they are both performed using computer vision algorithms. In situations when the camera is fixed and the backdrop remains constant, it is possible to detect items in the background using more straightforward methods. Aerial surveillance, on the other hand, is characterized by the fact that the target, as well as the background and video camera, are all constantly moving. It is feasible to recognize targets in the video data captured by an unmanned aerial vehicle (UAV) using the mean shift tracking technique in combination with a deep convolutional neural network (DCNN). It is critical that the target detection algorithm maintains its accuracy even in the presence of changing lighting conditions, dynamic clutter, and changes in the scene environment. Even though there are several approaches for identifying moving objects in the video, background reduction is the one that is most often used. An adaptive background model is used to create a mean shift tracking technique, which is shown and implemented in this work. In this situation, the background model is provided and updated frame-by-frame, and therefore, the problem of occlusion is fully eliminated from the equation. The target tracking algorithm is fed the same video stream that was used for the target identification algorithm to work with. In MATLAB, the works are simulated, and their performance is evaluated using image-based and video-based metrics to establish how well they operate in the real world.

## 1. Introduction

An example of this is the term “video,” which refers to a succession of images that are presented repeatedly. It permits the perception of human eyes to see the continuity of visual information in a continuous manner. In terms of the information content they convey, the two consecutive photos (referred to as frames) are very closely related to one another in terms of their composition. The visual hierarchy of abstractions that may be derived from the visual material can be found in this frame. Raw pixels are the first level of the hierarchy, and they include information on color and brightness, as well as other characteristics. When the picture is processed further, it is possible to get features, such as edges, lines, curves, and regions of high color intensity, among others [1]. A higher degree of abstraction allows for the merging of various traits, which results in the production of attributes (called objects). The interpretation of several things and their relationships is carried forth. According to temporal interpretation, the stages of a video are characterized as a frame, shot, and scene to express the hierarchical structure of a video in a more straightforward manner. The frame level of organization is the lowest level of organization in this hierarchical scheme. It may be required to split video footage into shots under certain circumstances. The term “shot” refers to a collection of photographs that represents a continuous sequence of events [2]. Continuous photographs are stitched together to form a single scene. Digital movies are created by combining photographs and films taken in a real-world context that include 3D objects in motion with computer-generated animation. When you see objects move, they are projected as a continuous sequence of pictures, which means that the intensities and colors of the images change as the things move. Actually, motion detection is the first step in the majority of video processing algorithms, and it is used to determine whether objects are moving by assessing the movement of their intensities or colors. It is possible to use the anticipated motion parameters for extra processing and analysis once they have been computed. Because of the temporal component of the video, however, significant increases in the quantity of storage, bandwidth, and computational resources are required [3]. Efficiency algorithms that make use of specific aspects of video, such as temporal redundancy, are required to decrease the need for complex processing and the requirement for more storage. Even if computer vision and human vision are both motivated by a similar purpose, they do not perform exactly the same functions. Human vision is fully reliant on the observer's point of view when it comes to perception. Every individual's experience with perception will be unique in its consequence. Computer vision relies on algorithms and the declarations that make up its components to function properly. Because of this, the result of the procedure is contingent on the computational framework that was used to develop it [4]. Surveillance, control, and analytical applications of computer vision may all be divided into three groups, according to their function. When it comes to any surveillance software, object detection and tracking are the most important components to consider. It is a noninvasive approach of observing and analyzing the motion patterns of objects in video with the goal of collecting information from the movie, and it is used in many different fields. For the purpose of governing the motion and, therefore, the visual system in control applications, certain requirements must be taken into account [5]. More information about analysis programs, which are often automated and used to diagnose and enhance the functioning of the visual system, may be found in the following section.

### 1.1. UAV-Based Aerial Surveillance

An unmanned aerial vehicle's (UAV) ability to conduct aerial surveillance has a broad variety of possible uses, including traffic monitoring in cities and highways, security guarding for significant events and buildings, and the identification of military targets, among others. It implements access control in restricted places, such as military bases, allowing for the restriction of unknown and undesirable movements in these regions [5]. Unmanned aerial vehicles (UAVs) may be used to conduct security reconnaissance, and they can also be used to ensure the safety of people. The movement patterns of cars on the highway or in congested traffic regions may be observed and recorded for later analysis [6]. The behavior of individuals may be watched noninvasively, allowing for close monitoring of the behaviors taking place in public gathering areas with a large number of people. In the course of identifying and tracking a target using an unmanned aerial vehicle, the issues that might arise are as follows:

- A 2D representation of a 3D object. As a result, a considerable amount of information is lost.
- It is possible that the objects may move in a complicated manner with varying velocity and acceleration.
- The low picture resolution induced by compression may result in poor quality data. The proposed work, shown in Figure 1, focuses on processing the video data collected from an unmanned aerial vehicle (UAV) to extract some information about the target, such as its size, direction, and description [7]. It is accomplished by the use of target identification and tracking algorithms. The method of predicting the temporal position of one or more items of interest in a video stream collected by a visual camera is known as video detection and tracking.

The aircraft will be controlled by a ground controller from a control station on the ground (GCS). The video will be provided from the UAV to the GCS in addition to telemetric data. The user initiates tracking by picking the item of interest from a list of options [8]. The target identification and tracking algorithm should take into account the needs and purpose for which it is being developed. In the case of an aerial platform, the key challenges that a video processing system would have to deal with include object identification, recognition, clustering, and variation in posture, equipment limits, and changes in the external environment [9]. When developing an algorithm, various elements of unmanned aerial vehicles (UAVs) must be taken into consideration. The height and surroundings are the most important considerations [10]. The UAV can fly at altitudes ranging from 50 to 1000 meters and at a maximum speed of 20 kilometers per hour. The unmanned aerial vehicle (UAV) may be operated at any time of day or night and in any weather condition. It is also necessary to examine difficult circumstances, such as those involving tiny items, obstructions, and drastic changes in the landscape [11]. During the course of the game, the target may enter and exit the field of vision several times. If there is any interference between the UAV and the GCS, noise will be added into the video stream, making it more difficult to identify, discriminate, and track the objects in the video stream [12]. The primary goal of the proposed project is to examine and explore different concerns and solutions related to surveillance footage taken by unmanned aerial vehicles. To determine the possibility of applying different video processing algorithms for aerial videos to extract some valuable information, this study was conducted [13]. This project involves the development and implementation of an aerial platform target identification algorithm and a target tracking algorithm that is suited for the dynamic environment. The aim of the proposed work is to develop target recognition and tracking algorithms using variety of data sets with varied environmental circumstances [14]. The main objective of the proposed work also includes the comparison of the performance with the existing algorithm.

The study is organized as follows: Section 2 is a review of the literature, Section 3 is a description of the proposed work's approach, Section 4 is an explanation of the experimental setup, and Section 5 is a discussion of the findings and analysis. Section 6 is divided into two parts: discussion and conclusion.

## 2. Literature Survey

Many research studies on mean shift tracking have shown that the method is resilient against overlap, occlusion, and nonrigid bodies, among other things. However, there are flaws in the monitoring of mean shifts [15]. For starters, the spatial relationship between the pixel and the target is no longer there. The algorithm then converges to false detection when the background and target have a color attribute that is similar to one another. These flaws are the consequences of using a simpler color histogram model to define the goal in the first place [16]. The tracking of the mean shift is based on the measure of similarity between two locations (Rubner et al. 2001) [17]. These dissimilarities are assessed based on the color and textural characteristics of the objects. In most tracking methods, the Bhattacharyya Coefficient (Aherne et al. 1998) [1] is used to calculate the measure. A variety of other distance measurements, such as the Euclidean measure, may also be used. Lee et al. [18] present a modified method to the mean shift algorithm for head tracking, which they call the modified technique. Whenever an item crosses beyond the border, the tracking algorithm is unable to locate the intended target [19]. The problem of convergence inside the border is resolved using a modified approach. A unique mean shift approach with an adaptive measure for tracking targets in FLIR image data was developed by Yin (2009) [20] and is described in detail below. In the first frame, the user sets the target's location by dragging a rectangle around it. For each target, numerous features are retrieved, and an adaptive selection measure is constructed based on the online feature ranking approach and the target's characteristics [21]. To adjust for motion on the moving platform, a technique known as block matching is used. It was hypothesized by Comaniciu et al. (2000) [22] that the mean shift tracking approach for real-time stiff objects will give higher tracking performance while requiring less sophisticated calculations. Direct projections into a new frame, on the other hand, cause a bias in the location estimate. As a result, Comaniciu and Meer (2002) [23] developed an improved version of the approach that incorporates feature space analysis. When the existence of a major feature is combined, it results in a high degree of tolerance-to-noise level exposure [24]. The features with lower levels of support are not recognized. As a result, just a small amount of critical information may be lost. It is possible to overcome the drawback of deleting a conspicuous feature by enriching the feature space with extra parameters from the input domain, as described above. It may also be prevented by the use of preprocessing processes [25]. In the kernel-based tracking technique, Comaniciu et al. (2003) [26] have made significant advancements in this area. The method performs well in the presence of camera motion, partial occlusions, target scale fluctuations, and clutter. It requires a complex filter model to prevent occlusions and clutter. The approach makes use of a set amount of bandwidth. In this case, Bradski's CAMShift method is used to address the problem (1998) [27]. The CAMShift successfully handles noise characteristics without the requirement for any specific filters to be used. Because the CAMShift approach is based only on color distributions, it is not possible to completely eradicate color-related sounds. Allen et al. (2004) [28] address this issue in a modified version of the CAMShift technique that uses quantized feature spaces to address the problem. The technique fails when the camera moves because it is based on a static backdrop model that is unable to appropriately depict [29] the changes in scenery as the camera moves. When the target's color is similar to that of the backdrop, the method fails as well, as previously stated. Stolkin et al. (2008) [4] developed an adaptive background candidate mean shift tracking strategy to deal with the problem of background similarity and similarity in candidate mean shift tracking [30]. The algorithm is resilient in the face of camera motion and pixels of identical hue for the backdrop and target [31]. Parameswaran et al. have devised a rapid way to mean shift tracking, known as the path assigned mean shift approach (PAMShift) (2008) [32]. Although the technique is quick, the bandwidth and kernel have been defined incorrectly in this case. It is as a consequence of this that targets are mislabeled as background and vice versa. Ju et al. propose and implement a fuzzy clustering-based solution to mean shift tracking, which they call “fuzzy clustering tracking” [33]. The approach is very durable and dependable. Clusters are generated by the usage of the membership function. With mean shift approaches, fewer mean shift iterations are necessary to reach the precise objective as opposed to conventional kernel-based strategies [34]. The RGB color model is the only one for which the algorithm is specified. Ning and colleagues suggest an adaptive technique to dynamically modify the size and orientation of the target. The method is only applicable to the ellipse and rectangle window functions, respectively.

It was published by Leichter et al. (2010) [35], who developed an innovative strategy that uses multiple reference histograms to update the target model. In this approach, multiple reference histograms are employed to update the target model [36]. As a result, this approach is computationally expensive, and thus, it is not suitable for real-time execution in the majority of scenarios. Azghani et al. (2010) [6] devised an intelligent technique for reaching convergence that was based on a genetic algorithm and used local search to achieve the aim. Although it is the case, the approach is bound by system-oriented limits and is not suitable for real-time applications. A Kalman filter may be used to update the target model to improve accuracy. However, even though using a Kalman filter to update the target model in each frame is computationally efficient, the process is time-consuming. Despite the several strategies used by Xiong et al. (2010) [37], enhancing the mean shift algorithm in complex settings in a real-world environment continues to be a tough undertaking. Using color and texture information, Bousetouane et al. (2013) [38] proposed a modified and adaptive mean shift tracking technique that incorporates color and texture information. The use of a new texture-based target representation that is based on spatial connections will be required moving forward. It is the degree to which two photos or frames are similar to one another in subsequent frames that determines the performance of tracking algorithms [39]. The distance between the two points is computed using one of the techniques listed below: [40] Bhattacharya, Hamming, Mahalonobis, Manhattan, or Euclidean distance are the terms used in distance calculations (Russel and Norvig 2003). An automated target discrimination system proposed by Chauhan et al. (2008) [41] has the potential to be employed in a wide variety of tracking applications, including guidance and navigation, passive range estimation, and automated target discrimination, to mention a few. The size, contrast, speed, and noise ratio of the tracker have an impact on its overall performance. As part of a quick evaluation strategy, the use of performance parameters, such as aiming point inaccuracy [42], duration of successful tracking, confidence indicator, number of tracking losses, and system reaction time for target tracking, is advised. According to Yang and colleagues (2010) [43], an approach that is more efficient than the previous one may be achieved by combining conventional algorithms with bandwidth adaptive algorithms. Identifying and tracking the target is accomplished by the use of background removal in combination with the mean shift target tracking technique [44]. A model update strategy based on an object kernel histogram was proposed, with the object kernel histogram serving as the basis. Only when the size of the targets is raised, does the approach become more robust to failure. Accordingly, Chen et al. (2011) [45] created a new similarity index for the CAMShift approach, which was utilized to compute pixel weights for the target model and candidate mode based on moments. Using aerial images, they demonstrated how to calculate the length and breadth of a car. While this is a kind of attribute, it may be any other type of characteristic, such as color, shape, or size. Next, they cut the photo into rectangles of the correct size, which they subsequently sew together to form the final product. Whenever a rectangle has a sufficient amount of foreground pixels, it is preserved as a likely candidate to be utilized as a target in the next Step [46]. The pixels of the candidates are shifted repeatedly using mean shift until they find a convergent location, at which point they are eliminated. A rectangle is joined with another rectangle if the overlapping area has a sufficient amount of foreground pixels. Until convergence has been attained, the merge procedure is repeated as many times as required. Although equivalent strategies may be implemented, one disadvantage of doing so is that the mean shifting methodology surpasses them in terms of performance. The foreground binary picture may be misclassified as numerous objects if there are errors in the foreground binary image, such as incorrectly partitioning large items, as seen in the following example. Specifically, a greedy algorithm explains how items are assigned to the anticipated ones and how things are assigned to one another inside the algorithm. In all of their experiments, they were able to achieve an almost perfect detection rate, according to their results. When dealing with challenges, such as occlusion, displacements, noise, image blur, background changes, and so on, they opted to depict their objects using the color histogram since it has been shown to be robust to appearance changes and to have a low degree of complexity. The primary disadvantages of employing color histograms are that no spatial information is provided and track loss may occur if there are obstacles with similar color combinations on a track. As a consequence, it is proposed that spatial information be added to target representation while keeping the favorable properties of the color histogram to make it more robust. The usage of a multiple kernel representation in combination with a particle filter is used to achieve this. To divide the object, which is contained inside a rectangle, into several kernels, each of it is weighted differently, depending on how essential it is in relation to its location within the object. PF is used to overcome short occlusions and interference caused by background noise and other sources of interference. Once a set distance between the smallest particle and the object has been exceeded, object loss or full occlusion are considered possibilities. In this paper, we provide a multipart color model that was tested on eight different color spaces covering three different modern trackers. The PF tracker, MS tracker, and Hybrid tracker were the names given to these trackers, and they were all tested on the MS tracker (HT). Each of the eight color spaces has its own set of color histograms, which are computed. As the RGB color space surpasses the other color spaces without compromising a single track, the authors reach the conclusion that it is superior. As a consequence, the RGB color space has been chosen for use. In addition to size and orientation, the existing technique recommends two forms of multidimensional histograms: one that adds color and texture information about the object in each frame, and another that does not integrate such information. Because of their high degree of directionality and ability to produce a flat surface, they are widely used. When used in conjunction with the contourlet transform, the histogram approach provides very robust rotation and deformation features. It has been proposed to use an adaptive contour feature (ACF) for human detection, which is composed of the number of grain granules in the picture in oriented space and is meant to be robust to changes in the image.

Manual identification and tracking is a time-consuming endeavor that requires patience. In this project, techniques for automatic and semiautomated detection and tracking are being employed to gather information. When using these tactics, it is common to maintain a model that is tied to the spatial relationship between many variables, such as motion, color, and edge. Videos may be separated into two groups based on how they are segmented: spatial segmentation and temporal segmentation. A digital image segmentation approach is used to create the spatial technique. Digital image segmentation divides an image into portions of two or more levels of detail, which may be done locally or globally, depending on the application.

## 3. Methodology of Proposed Work

V2V communication has the potential to serve as a data-sharing platform, increase driver assistance, and enable the development of active safety vehicle systems. Driver aid is supplied by cooperative communication among cars, which allows information or warning messages to be broadcast and/or shared in an adaptive manner for the driver.

It may be further tailored to meet the needs of certain groups of individuals in the community, such as senior citizens driving. V2V communication includes features, such as lane maintaining, steering control, parking assistance, obstacle recognition, intervehicle spacing, and driver/vehicle exchange of optional/useful information while traveling along the same route.

Vehicle-area-network communication may be accomplished through a wireless connection, which can provide wireless LAN localization, among other things. When driving, automobiles may pick up on a variety of wireless signals, including GSM, cell tower signals, FM-AM radio transmissions, radar signals, GPS signals, and wireless LAN signals, among others. Specific differential GPS techniques have gained popularity in recent years for determining more precise coordinates for localization. In a wireless LAN, a large number of access points broadcast beacons on a regular basis. When a vehicle enters a wireless LAN-enabled region, the vehicle may get information from beacons, such as the service-set identification (SSID), MAC address (BSSID), signal strength, and vehicle's location with respect to the access point. Aside from that, it is possible to determine the vehicle's speed by examining the difference in signal intensity distribution across different mobilities.

This platform allows for the usage of cellular/Wi-Fi devices for both short- and long-range intervehicle communication. Wireless connections that meet the power/bandwidth requirements, such as GPRS used in 3G cellular communication systems, 4G ultra-high-speed mobile broadband, such as long-term evolution (LTE) mobile broadband, and mobile Wi-Fi hotspot, provide standard connections for multiple vehicles and their associated devices.

Various applications need different sensors, processing units, and, in some cases, even actuators are to be implemented. On the market, there are already a number of goods, such as a lane-passing alert in the Mercedes-Benz W163-M class, brake assist/navigation link in Toyota, tire sensors in Fiat, blind-spot recognition in BMW, and collision mitigation brakes in Honda, among other things. This field, on the other hand, is still in its infancy. In reality, the sky is the limit when it comes to creative systems and devices that are affordable and meet the needs of consumers.

At the moment, cooperative or cognitive communication among automobiles is still in its early stages. The objective is to make data interchange easier and to build a network that is very informative. A heterogeneous network architecture that enables wire-speed, robust, seamless, and secure communication is currently being developed, despite the fact that the LTE-connected car initiative (www.ngconnect.org) and the iDrive system with Internet connectivity (www.bmwblog.com) were only recently introduced.

There are other unanswered concerns that must be addressed, including the following: what information can or cannot be broadcast or received by a single vehicle and how to structure packets for more effective delivery. This kind of distribution is particularly difficult because of the limited amount of time (on the order of a few seconds at the most) when vehicles are within the access range of one another.

Communication from a vehicle to the cloud (V2C) is discussed in detail in section B.

Many valuable applications are made possible by vehicles connecting with a broadband cloud, such as, for example, a monitoring data center in a vehicle-area-network environment. Vehicles may be able to communicate via wireless broadband technologies, such as 3G and 4G (HSI).

High-speed 4G mobile broadband technologies, such as LTE and 802.16m-based WiMAX, which may achieve download speeds in the excess of 100 Mbps, will be highly sought after in the future. This form of communication will be particularly beneficial in network fleet management applications, such as active driver assistance and vehicle/driver tracking, among others. Furthermore, the cell phone device itself might be utilized as a gateway in this platform to transmit and receive data between central monitoring data centers linked to the broadband cloud [47] and other data centers.

The following are two ways in which V2C networks might give relevant information:

The first type of data is outgoing data, which may include: (a) vehicle-centric information, such as speed, global positioning/routing, device functionality, and performance, and (b) driver-centric information, such as driver-specific behavior (e.g., drowsiness, length of continuous driving), audio/video, and so on. The second type of data is incoming data. All of this information may be transferred to a central monitoring server/system for additional analysis and storage if desired by the system administrator.

Data comes from a central office, which may involve receiving data from a central office for different communications with the driver and/or the vehicle system.

It is the first critical stage in information extraction for computer vision applications, such as people tracking, video surveillance, traffic monitoring, and semantic annotation of videos, among others, when a moving object is detected and tracked in a video stream. There should be particular features in the algorithms used for object identification and tracking in these applications that set them apart from the other techniques of identifying and tracking objects.

The following attributes may be found in abundance: flexibility in a number of situations (indoors and outdoors) and adaptability in a variety of lighting conditions are the advantages of this technology. Having the capacity to execute rapidly and adapt to a wide range of scenarios should be seen as essential requirements that must be met. The tracking of an item becomes more trustworthy (the same object may be recognized more consistently from frame to frame if its shape and location are accurately identified) and more efficient when precise form and position detection is used. Input video data is received from an unmanned aerial vehicle (UAV) via satellite. By deploying the UAV in a real-time environment, a collection of aerial films with a range of circumstances and qualities may be collected and then used as input data for the algorithms that have been developed to analyze the data that has been gathered and collected. The user has the option to designate the target in the video frame by dragging the mouse over it. The existence of a certain target in the background noise may be detected using a running Gaussian background subtraction technique (RGBS). The suggested technique is compared against many existing methodologies, including temporal frame differencing (TMF), running average background subtraction (RABS), and temporal median filtering (TMF). The target tracking algorithm is given the exact same video as the source tracking algorithm to work with. The adaptive background mean shift tracking (ABMST) technique, which has been proposed and developed, is used to continuously monitor the target of interest in real time. The proposed approach is compared to the traditional mean shift tracking technique (TMST) and the continuously adaptive mean shift technique (CAM Shift) to show its advantage in terms of efficiency over the other two techniques. A flowchart of the work process is shown in Figure 2.

### 3.1. Detection of Targets in Video Frames

When it comes to surveillance applications, detecting moving objects from a video stream is a basic, yet crucial operation. When it comes to the identification of moving objects, background subtraction is a general strategy that compares each received video frame with a previously produced backdrop model that is supposed to be the standard. It is regarded to be an element of a moving object when a pixel in the current video frame deviates considerably from the reference frame. In the case of airborne surveillance, the algorithm must be able to react to a variety of challenges, such as changing lighting conditions, a cluttered backdrop, cast shadows, snow, and fog, among others. Furthermore, to ensure real-time practicality, the technique should be computationally efficient and have minimal memory needs.

To put it simply, background subtraction is the process of subtracting a picture from a reference image. The background scene in this reference photograph is a model for the scenario in the foreground. In the fundamental stage shown in Figure 3.2, background modeling, thresholding, and the operation of subtraction are performed.

- The backdrop modeling process entails the creation of a reference picture that serves as the background representation.
- The determination of the threshold value for the subtraction operation is carried out at the threshold selection stage.
- During the subtraction stage, the pixels are classified as either being in the background or being a moving item.

Temporal or neighboring frame differencing is the most fundamental approach for distinguishing the backdrop from the target in video footage. It entails the removal of subsequent frames to construct a backdrop model for the scene. It makes the assumption that the first frame is the background model and subtracts the subsequent incoming frame from the presumed background model. The resulting frame is used to create a new backdrop model, which is then compared to the previous frame. This technique is repeated until a total of “n” frames of video data are collected.

The input video sequences are arranged as frames, which are represented as g1, g2, g3 … .gm , with *m* frames. Let the initial sequence ID be represented as *g*_*i*_, with the background model *c*_*i*_.

(1) $$\begin{array}{c} c_{i=}g_{i}\text{where }i=1,\\ g_{i+1}-g_{i}=c_{i}+1,\\ i=1,2\ldots m. \end{array}$$

where *g*_*i*_ is the *i*^th^ frame and *g*_*i*_ + 1 is *i* + 1^th^ frame.

The update g_i_ is obtained by subtracting the resultant background model c_i_ from frame f_i._

(2) $$\begin{array}{c} g_{i}-c_{i}=g_{i}. \end{array}$$

### 3.2. Running Average Background Subtraction

A technique known as running average background segmentation, also known as adaptive mean background subtraction, involves subtracting subsequent frames, depending on the background model and learning rate *i*, which is set at one second. Based on the mean intensity value of the background model developed for a total number of *n* frames of the input video, the thresholding procedure is carried out.

The first frame of the input video is assumed as background model c_i_ initially.

(3) $$\begin{array}{c} c_{i}-g_{i},i=1. \end{array}$$

To create the final background model ci + 1, the difference between the frame f_i_ and the previously assumed background model b_i_ is blended along with a proportional fraction referred to as the tuning factor (see Figure 1). The value of a determines the amount to which the two frames' contributions to the final background model are removed to construct the final background model. In the range of 0 to 1, the value of *f* must be used.

(4) $$\begin{array}{c} bi+1=afi+\left(1-a\right)bi. \end{array}$$

The update g_i_ is obtained by subtracting the background model *b*_*i*_ + 1 from the subsequent frames f_i_.

(5) $$\begin{array}{c} gi=fi-bi+1. \end{array}$$

### 3.3. Tuning Factor Optimization

The optimization of the tuning factor is an extremely crucial phase in the background modeling and updating process. Although each background layer is considered as neighbourhood pixels, active features can be calculated by increasing the neighbourhood pixels, and the motion distortion can eliminate extra noise. The amount of time spent creating the backdrop model is significantly reduced as a result of this. As a result, an ideal value that is applicable to all aerial platform scenarios is required. The optimization process is carried out on the premise that the statistical characteristics of the item vary significantly from those of the background.  Figure 3 represents the angle representation.

When it comes to the backdrop picture, the anticipated RGB color value for pixel 'j' may be calculated as follows:

(6) $$\begin{array}{c} \underline{\underline{F_{i}}}=\left[F_{Y}^{i},F_{G}^{i},E_{b}^{i}\right]. \end{array}$$

Generalizing the expectation parameter for *n* pixels,

(7) $$\begin{array}{c} \underline{\underline{F_{i}}}=F\left\{Y_{i}\left[m\right]\right\},1\leq m\leq M. \end{array}$$

The line OE is the expected chromaticity line. The RBG intensity value of the pixel “*i*” is as follows:

(8) $$\begin{array}{c} \underline{\underline{K_{i}}}=\left[K_{\mathbb{R}}^{i},K_{\epsilon }^{i},K_{B}^{i}\right]. \end{array}$$

There is a scale in the brightness distortion that makes the observed color closer to the intended chromaticity line. It may be represented by the symbol *σ*(*α*_*i*_).

(9) $$\begin{array}{c} \left.\frac{\sigma }{i}\;={\left(I-\sigma E\right)}^{2}.\right.. \end{array}$$

Compute the distortion of *Y*_*i*_[*n*] from its mean *E*_*i*_ by considering the orthogonal distortion parameter *σ*_*i*_(*m*).

(10) $$\begin{array}{c} \sigma_{i}\left(m\right)=\left(Y_{i}\left[m\right]-F_{i}\right)V_{y}. \end{array}$$

*V*_*y*_ is the unit vector in the *Y* axis, and *α*_*i*_(*n*) is the brightness parameter. Thus, the factor *a* for RGB space is defined as follows:

(11) $$\begin{array}{c} \sigma S\left(m\right)=\frac{Y_{i}^{R}\left(m\right)-F^{R}}{\sigma_{i}^{R}}, \end{array}$$

(12) $$\begin{array}{c} \sigma_{2}\left(y\right)=\frac{y_{i}^{\alpha }\left(y\right)-2/4}{c^{2}}, \end{array}$$

A conversion from RGB to HSI color space is necessary because of the significant correlation between the colors in the RGB spectrum. Specifically, equations (9)–(11) are normalized.

(13) $$\begin{array}{c} j=m\left\{b_{\Sigma }b_{a},b_{a}\right\}. \end{array}$$

*j* is the intensity value in the HSI space that includes the majority of the information for the processing operation. *H* and *S* values are automatically deleted. As a result, the ultimate turning factor “*b*” is calculated as follows:

(14) $$\begin{array}{c} b_{\gamma }\left(\pi \right)=\frac{y_{i}\left(n\right)-F_{j}}{\pi_{i}}. \end{array}$$

A value of 1 indicates that the brightness of the sample panel is identical to the brightness of the reference panel. A value less than one indicates a fair difference in brightness between the two panels under consideration.

Because n is an optimal parameter, its value may be any number between 0 and 1 for both static and dynamic ground models. Four videos are utilized in the analysis, and each video has 100 frames that are taken into consideration. Pixels are examined in each frame, with 500 pixels being evaluated at random places and their intensities being collected for processing. The mean, standard deviation, and variance of the pixel values are calculated using statistical calculations based on the data taken into consideration. The turning factor is calculated on the basis of these three criteria, and the results are displayed in Table 1.

V2V networks should be established in accordance with certain standards that specify the communication architecture, protocols, messaging, administration, hierarchy, and other aspects of the networks. This section provides an overview of the most important VAN standards.

- IEEE 802.11p: the IEEE 802.11p standard draught, which is currently in active development with a planned release date of November 2010, is an amendment to the IEEE 802.11 standard. It is still in the early stages of development. IEEE 802.11p is a wireless access in-vehicle environments (WAVE) standard that is intended to enable intelligent transportation systems (ITS) applications [33] by providing wireless access in vehicular contexts. This standard specifies the vehicle-to-vehicle (V2V) and vehicle-to-infrastructure (V2I) communication protocols for high-speed vehicles and is primarily concerned with design difficulties at the physical (PHY) level. In the United States, it is accomplished by the use of dedicated short-range communications (DSRC) at 5.9 GHz, which corresponds to the licensed ITS band of 5.85–5.925 GHz.
- IEEE 1609: the IEEE 1609 standard [35], which is an upper layer standard on which the IEEE 802.11p standard is based, is a ubiquitous vehicular communication standard that allows for communication across various automotive suppliers and manufacturers. The IEEE 1609 standard family comprises a set of WAVE-related specifications. It specifies the architecture, organizational/management structure, communication model, security measures, and physical access requirements for a system. As a whole, these characteristics make it possible to use secure V2V and V2I wireless communication in a wide range of applications, such as traffic management, active safety services, automated tolling, and so on.

Our fundamental belief is that an efficient in-vehicle platform increases the active features of vehicle area networks. Vision-based tools and sensors are used to gather critical information about the driver, the vehicle, and the car's surroundings on this platform.

When it comes to gathering crucial information about the road and surrounding environment, cameras are a low-cost alternative. Additionally, they are completely noninvasive and visible to the driver. Furthermore, cameras pointing outdoors may be universally accepted since there would be no fear of privacy being violated. If there is sufficient infrastructure on the road, data from the road might potentially be captured using vision-based techniques, such as cameras or sensor arrays. Image processing methods (e.g., MATLAB or bespoke software modules) may be utilized on this platform to extract important information and alert or aid the driver in potentially dangerous situations.

Vehicle data collecting might be accomplished by sensor technology that is completely invisible to the driver. Sensors would record changes in speed, pressure, and sequencing of the brake and gas pedals, and the shifting pattern of the steering-wheel angle, among other things. Eye closure/blink rate, yawn/chin-drop are the examples of physiological data that may be collected by the driver's camera. Other physiological signals such as heart rate, EOG, and other signals can be collected through sensors.

When it comes to in-vehicle processing, embedded microprocessors are required, and FPGA prototype units may be used for interfacing and specialized peripherals. After gathering photos or sensing data from the in-vehicle sensors, it is necessary to conduct behavior analysis to determine the presence of any anomalies. The results of the behavior analysis can then be sent to the following parties: (1) the driver (for example, an early warning of a fast-approaching car from behind), (2) a monitoring station (for example, fleet management), and (3) sharing among users (for example, road status data exchange among vehicles in the immediate vicinity).

According to Table 1, the average tuning factor for videos 1 to 4 is 0.602, 0.507, 0.498, and 0.528 using the method adaptive gaussian background subtraction. The tuning factor in its entirety is around 0.53. Thus, the value may vary between 0.5 and 0.6 to ensure effective segmentation.

### 3.4. Target Tracking

Target tracking is a technique for following single or numerous objects throughout the course of a series of frames. Tracking may be performed in either a forward or reverse direction. Mean shift tracking is a form of forward tracking. It makes an estimate of the object's location in the current frame based on the previous frame. It is a gradient ascending strategy that creates a histogram model of the visual area to be monitored. It extracts the density function's local maxima from the data samples. Mean shift tracking is a nonparametric, real-time, user-interfaced, kernel-based tracking technology that enables precise target localization and matching without the need for a costly search. It operates by iterative passion. It calculates the mean shift value for the current pixel location and shifts to the new position with the mean shift value, continuing until the requirements are satisfied.

In this section, we create a kernel function that determines the distance between the sample points considered and the mean shift point.

Mean shift tracking is an important tool in the field of target tracking because of its stability and computational economy. Classic mean shift tracking, on the other hand, is predicated on the premise that the target and backdrop are vastly different. Aerial footage, on the other hand, makes it impossible to tell the difference between the background and the target.

As a consequence, the old approach is unable to adjust to dynamic changes and consequently fails.  Figure 4 illustrates the notion of mean shift clustering.

The accuracy of mean shift tracking is dependent on the production of a candidate model that is compared against the target's location in incoming frames.

**Case 1 .**

The present location is a destination (vehicle A in Figure 5).

**Case 2 .**

Although the location is not a target, it shares the target's color attributes (vehicle B in Figure 5).

**Case 3 .**

The present place is not a goal and has no resemblance to it (vehicle C in Figure 5).

The mechanism for establishing the background position is determined by the preceding frame's data. The first frame identifies and models the target. The following frame creates a candidate model. The window is moved according to the difference between the target and candidate models. The new location is determined using the scale and orientation of the centroid position in the CAM shift approach. It is appropriate only when the frame movement is linear and steady.

There will be shear and angular displacement in the footage shot by unmanned aerial vehicles. Thus, the altered location of a single point in the incoming frame does not aid in the precise localization of the target. A complete representation of the target's backdrop is needed, including the distance and angle for each pixel in the given target window.

Assume that the target model has a center of gravity of “y.” The target model's bin size, area, and color scheme are established. The initialization is carried out using the strategy kernel, as seen in Figure 6

(15) $$\begin{array}{c} F\left(y\right)=\left\{\begin{array}{c} 1-y^{2},\;\text{if }0\leq y\leq 1,\\ 0,\text{ otherwise}. \end{array}\right. \end{array}$$

## 4. Results and Analysis

Frame-based performance indicators are grounded in reality. Ground truth often contains abstract data (location, size, and type) that may be compared to the extracted video frame observations. Bashir and Porikli discuss the metrics (2006). The ground truth must consist of a circle or bounding box, indicating the target's position. Precision rates give the target a positive value. Classification of data derived from the obtained result.

The examination of ground truth is predicated on four fundamental terminologies: true positive (TP), false positive (FP), true negative (TN), and false negative (FN).

True positive: the ground truth and the result agree on the target's existence, and the result's bounding box and the ground truth correspond. True negative: the target's absence is confirmed by the ground truth and the final result. False positive: tracker identifies an item, however, the ground truth does not include any objects or no system objects fall inside the bounding box of the ground truth object.

False negative: the ground truth detects an item, however, the tracker does not.

On the basis of these metrics, the following parameters are evaluated: completeness (CS), false alarm rate (FAR), similarity (SS), and accuracy (ACC) for traditional mean shift tracking, continuously adaptive mean shift tracking (CAMS), and the proposed adaptive background mean shift tracking in terms of the total number of frames (TF). For each video dataset, the findings are tabulated and the corresponding graphs are shown.

(16) $$\begin{array}{c} \text{Completeness}\left(\text{CS}\right)=\frac{\text{T}}{\text{T}+\text{FN}},\\ \text{False Alarm Rate}\left(\text{FAR}\right)=\frac{F}{T+F},\\ \text{Similarity}\left(\text{SS}\right)=\frac{T}{T+K+KN},\\ \text{Accuracy}\left(\text{ACC}\right)=\frac{\text{T}+\text{IN}}{\text{IF}}. \end{array}$$

The length of successful monitoring (DOST) is a metric that is assessed based on the ratio between the number of frames in which the target is tracked successfully and the total number of frames in which the target is visible (or visible frames).

(17) $$\begin{array}{c} \text{OST}=\frac{\text{No}.\text{of seconds target is successfully tracked}}{\text{No}.\text{of seconds in video}}. \end{array}$$

The tracking rate (TR) is obtained by dividing the total number of input frames by the number of frames that were accurately tracked. In this section, the results of frame-based performance metrics are determined for the classic mean shift approach, the continuously adaptive mean shift technique, and the suggested adaptive background mean shift technique. For the sake of simplicity, the metrics are shown as a graph.

### 4.1. Implementation of Target Detection Algorithms

In this section, the results of the proposed running Gaussian background subtraction technique for target detection for 10 different video data is shown and discussed as a comparison with temporal median filtering technique, running average background subtraction, and traditional frame differencing technique.

### 4.2. Target Detection Results for Dataset 1

There is a target to be tracked (a cow) in video data 1, and the animal moves randomly. Indeterministic movement of the target is seen. It is altering its form, direction, and speed in relation to the goal specified. Angular footage filmed from a low height at Kovalam beach in Chennai, India, with an experimental bias is shown in this video.  Table 2 list the characteristics of the video.  Figure 7(a)–7(e) (a, b, c, d, and e).

Initial stages are characterized by high PSNR values for detecting approaches since the UAV is hovering and the target is also motionless throughout this time period. After a few frames, the target begins to move, and the UAV begins to follow the target as well. Because of the mobility of the sensor and the target, ego noise is generated, and the efficiency is reduced to a certain level. Despite the fact that the value of metrics is decreasing, it remains greater than other techniques. Plotting the PSNR in Figure 8 illustrates the fluctuation in measurements across time. Figures 8–12 represent the performance metrics of the proposed work.

The performance metrics for adaptive background mean shift tracking method are greater than those for traditional mean shift tracking and continuously adaptive mean shift tracking technique, as shown in the above data. The tracking algorithm on a moving platform has better efficiency than previous methods.

The following are the interpretations based on the findings:

- The backdrop model of the specified target has a significant role in the target tracking algorithm's performance.
- When the backdrop is smooth, the tracking rate is greater, however, when the background is crowded, the tracking rate is lower.
- The tracking algorithm is unaffected by changes in light or partial incursions because of the tracking method.

It is not affected by changes in orientation, size, or altitude when using the ABMST approaches.

## 5. Conclusion

As a result, effective algorithms for target recognition and tracking in aerial video streams are developed and put into action by researchers. The algorithms are being designed to be suitable for applications that operate in a strict environment, such as aerial surveillance. The preceding findings demonstrate that the value of PSNR for the running Gaussian background removal is comparable to that of other approaches when compared to other techniques. The greatest PSNR value is in the region of 65, which occurs during the early phases of background noise. It is because of the fact that at the beginning of the process, when the backdrop model is updated, it will seem more like the sample frame. However, when the number of frames grows, the new model will be based on the prior model and the current frame. As a result, there is a modest deterioration in the definition of the backdrop model. The MATLAB program is used to mimic the works that were completed for the thesis. The simulation work is primarily concerned with addressing the issues that arise during the processing of aerial footage. Background subtraction approaches may already be realized in hardware by the use of embedded processors and reconfigurable processors, among other technologies. However, there is a constraint in that they are implemented with a static backdrop. As it is equivalent to previous approaches in terms of efficiency, the adaptive Gaussian background segmentation-based detection methodology is possible for real-time use while maintaining its effectiveness. Because of the fixed values of adaptation, the processing time will be faster than that of the running average approaches. So far, the mean shift tracking approach has been deployed in real time for applications, such as face identification and traffic monitoring. The backdrop of the working platform is stationary, while the target is shifting. While the suggested adaptive background mean shift tracking approach is not as fast as classic techniques, it is viable in real time and provides a suitable solution to ego motion problems. To be used in UAV applications, the algorithm may be put onto a chip and installed on the drone's board as a payload. It is possible to do the processing while the UAV is in flight, and the results are relayed to the ground control station [48].

## Figures and Tables

**Figure 1:** Model for collecting input data.

**Figure 2:** Work flow diagram.

**Figure 3:** RGB color space of a pixel “*i*”.

**Figure 4:** Concept of mean shift clustering.

**Figure 5:** Target definition: mark A denotes the target, B denotes a mark that is not the target but has comparable attributes to the target, and C denotes a mark that is completely distinct from the target.

**Figure 6:** Proposed shift tracking algorithm.

**Figure 7:** (a) Initial frame for input video 1. (b) Background model of sample frame 4. (c) Background update of sample frame 4. (d) Background subtraction of sample frame 4.

**Figure 8:** PSNR for dataset 1.

**Figure 9:** False alarm rates for target-tracking techniques.

**Figure 10:** Accuracy measure for target-tracking techniques.

**Figure 11:** Duration of successful tracking of target-tracking techniques.

**Figure 12:** Tracking rate of target-tracking techniques.

**Table 1:** Optimization of tuning factor.

Video	Mean	Variance	Standard deviation	Tuning factor
Video 1	0.8147	0.9134	0.2785	0.602
Video 2	0.9058	0.6324	0.5469	0.507
Video 3	0.1270	0.0975	0.9575	0.498
Video 4	124.955	1786.522	42.267	0.528

**Table 2:** Target detection metrics for dataset 1.

	LM	CM	SM	MSSIM	MSE	PSNR	DR
TFD	2.735	43.69	62.23	0.941	0.945	0.068	0.061
RABS	2.413	44.32	65.57	0.982	0.985	0.072	0.070
TMF	2.159	44.81	67.21	0.985	0.982	0.075	0.072
RGBS	1.950	45.23	75.41	0.999	0.997	0.082	0.082

## Data Availability

The data that support the findings of this study are available on request from the corresponding author
